# Discovery of New Therapeutic Targets for Osteosarcoma Treatment Based on Immune-Related lncRNAs in the Tumor Microenvironment

**DOI:** 10.1155/2022/3113857

**Published:** 2022-04-26

**Authors:** Ribin Fu, Xiaofang Hong

**Affiliations:** ^1^Department of Joint Surgery and Sports Medicine, Zhongshan Hospital, Xiamen University, Xiamen 361004, China; ^2^Department of Stomatology, Zhongshan Hospital, Xiamen University, Xiamen 361004, China

## Abstract

**Background:**

Long noncoding RNAs (lncRNAs) play an important role in osteosarcoma development, but their role in the tumor microenvironment (TME) is not fully understood. This study associated lncRNAs with immune-related genes and explored the mechanism of lncRNAs in osteosarcoma progression.

**Methods:**

Unsupervised consensus clustering was applied to construct immune subtypes based on immune-related lncRNAs identified by Pearson's correlation analysis. A series of functional analysis was performed to reveal the links among lncRNAs, immune subtypes, TME, and osteosarcoma prognosis.

**Results:**

We identified two immune subtypes C1 and C2 showing distinct overall survival. ECM-receptor interaction pathway was more activated in C2 subtype, while immune response pathways were more enriched in C2 subtype. Differential TME and response to chemotherapeutic drugs were observed between the two subtypes. Four metagenes of costimulation, cytolytic activity (CYT), immune score, and STAT1 were differentially enriched in the two subtypes. Based on 26-paired lncRNAs, we constructed a 4-paired lncRNA prognostic signature for predicting prognosis of osteosarcoma prognosis.

**Conclusions:**

This study focused on immune-related lncRNAs and TME, showing the possible role and mechanisms of lncRNAs in tumor growth and metastasis. ECM may be the new therapeutic target for treating osteosarcoma, and 26-paired lncRNAs could serve as a basis for further studying the mechanisms of CYT and STAT1 in immune response, cancer cell proliferation, and migration. The two subtypes and prognostic signature could promote the design of personalized osteosarcoma treatment.

## 1. Introduction

Osteosarcoma, which is the most common bone malignancy derived from mesenchymal cells, frequently occurs in children and young adults. About 20% osteosarcoma patients will develop metastasis of which pulmonary metastasis accounts for nearly 80% of all metastatic cases [1, 2]. 5-year overall survival of metastatic osteosarcoma patients and recurrent patients greatly varies but is still lower than 30% [2]. Although adjuvant and neoadjuvant chemotherapy and aggressive surgery are currently employed as the standard for treating osteosarcoma, approximately 30-40% patients still suffer from relapse [1, 3].

In recent years, immunotherapy, especially immune checkpoint inhibitors, has emerged as a new approach to treating various cancers, and a series of clinical trials show favorable outcomes [4, 5]. However, the results of clinical trials using immune checkpoint inhibitors such as ipilimumab and pembrolizumab for treating osteosarcoma are disappointing [6, 7], which may be due to suppressed immune response generated by tumor microenvironment or a lack of neoantigens. Wu et al. compared the level of immune infiltration among different cancer types and found that a majority of osteosarcoma patients show less immune infiltration than other cancer types, which could explain a low response to immune checkpoint inhibitors [8]. In addition, three immune subsets of osteosarcoma with different levels of immune infiltration were defined, and close correlation between genomic alternations and immune suppression was found [8]. However, to fulfill an effective targeted therapy, the mechanism of osteosarcoma development and progression should be further understood.

It has been previously demonstrated that aberrant expression or regulation of long noncoding RNAs (lncRNAs) are associated with cancer development [9]. For example, DANCR and TUG1 upregulated in osteosarcoma tissues can enhance migratory potential and invasion of osteosarcoma cells [10, 11]. LINC00588 is a tumor suppressor that hinders tumor cell proliferation, migration, angiogenesis, and epithelial-mesenchymal transition (EMT) through acting as a ceRNA for miRNA-1972 in osteosarcoma [12]. In oncogenic pathways such as PI3K/AKT and WNT signaling pathways, lncRNAs play a modulatory role in the activity of these pathways [13–16]. Moreover, lncRNAs secreted from tumor cells are critical molecules for mediating cell-cell communications in tumor microenvironment (TME), thereby providing a tumor-supportive microenvironment [17, 18]. T. Zhang et al. constructed a signature of 12 immune-related lncRNAs and 3 immune-related genes for predicting osteosarcoma prognosis [19]. Therefore, lncRNAs can serve as predictable biomarkers for indicating prognosis or promising targets for personalized therapies.

In this study, we applied a paired lncRNA strategy to identify two immune subtypes and constructed a 4-paired lncRNA prognostic signature for osteosarcoma. Further integrative analysis discovered the pivotal role of lncRNAs in TME and osteosarcoma development. The findings paved an important step for searching new lncRNA-based targeted therapies and allowed an early identification for osteosarcoma patients with high-risk metastasis.

## 2. Materials and Methods

### 2.1. Data Information and Preprocessing

RNA-seq data and clinical information of osteosarcoma samples were downloaded from TARGET database (https://ocg.cancer.gov/programs/target/data-matrix). The samples without clinical information, survival time, or survival status were excluded. We use R software package hgu133plus2.db to convert Ensembl ID into gene symbol. Median expression level was selected when one gene had multiple gene symbols. After data preprocessing, 84 osteosarcoma samples (55 alive status and 29 dead) were retained, including 47 male samples and 37 female samples. The workflow of this study was shown in Figure 1.

### 2.2. Identification of Immune-Related lncRNAs

Immune-related genes were obtained from ImmPort database (http://www.immport.org, Release 42, January 2022). Latest gene transfer format (GTF) file came from GENCODE (https://www.gencodegenes.org/, GRCh38.p13). mRNA and lncRNA expression profiles of osteosarcoma were distinguished by GTF file. Then, Spearman's correlation coefficients were calculated between each immune-related gene and each lncRNA. Finally, 42 immune-related lncRNAs were screened under the conditions of correlation coefficient > 0.4 and false discovery rate (FDR) < 0.05.

### 2.3. Pairing of Immune-Related lncRNAs

Loop pairing was implemented to pair immune-related lncRNAs. Zero or one matrix was constructed based on the assumption defined as follows: lncRNA A and lncRNA B were paired, and their expression difference was defined as C; C was defined as 0 when lncRNA A expression was lower than lncRNA B; otherwise, C = 1. In this way, 375-paired lncRNAs were included with the condition that the proportion of C = 1 was 40%-80%.

### 2.4. Consensus Clustering for Identifying Molecular Subtypes

Paired lncRNAs related to osteosarcoma prognosis were identified by univariate Cox regression analysis using coxph function in survival R package. Consensus clustering in ConsensusClusterPlus (v1.48.0) R package was conducted under parameters of reps = 100, pItem = 0.8, pFeature = 1, distance = ^“^spearman^”^, and clusterAlg = ^“^pam^”^ [20].

### 2.5. Immune Analysis of Molecular Subtypes

GSVA R package was used to perform single sample gene set enrichment analysis (ssGSEA) for calculating enrichment score of 22 immune cells and 13 immune metagenes [21, 22]. Each immune metagene contained a series of immune-related genes. Immune score was calculated by ESTIMATE method [23]. 47 immune checkpoints obtained from the previous study were included to further assess tumor microenvironment [24]. Log2 (gene expression + 1) was defined to analyze the expression level of the 47 immune checkpoints.

### 2.6. Analysis of KEGG Pathways and GO Function

In function analysis of molecular subtypes, we first identified differentially expressed genes (DEGs) with |fold change (FC)| > 1.5 and *p* < 0.05 by limma R package [25]. Then, WebGestalt R package was performed to annotate Kyoto Encyclopedia of Genes and Genomes (KEGG) pathways and Gene Ontology (GO) terms [26].

Spearman's correlation analysis was conducted to calculate each correlation coefficient between each paired lncRNA and each mRNA. Correlation coefficient > 0.3 and *p* < 0.05 were the criteria to screen genes significantly associated with paired lncRNAs. Then, WebGestalt R package was used to annotate KEGG pathways and GO terms.

### 2.7. Construction of a Prognostic Model

A total of 84 osteosarcoma samples were divided into training cohort and test cohort with a ratio of 1 : 1 for 100 times of random sampling. coxph function in survival R package was applied to perform univariate Cox regression analysis for detecting immune-related paired lncRNAs associated with prognosis (*p* < 0.05). Least absolute shrinkage and selection operator (LASSO) Cox regression analysis in glmnet R package was employed to reduce the number of variables (paired lncRNAs) [27], and 10-fold cross validation was used to construct models. Next, step Akaike information criterion (stepAIC) in MASS package was used to further optimize the model [28]. The least number of variables was remained to acquire enough fitting degree. The coefficient of finally remained paired lncRNAs was calculated by multiple Cox regression analysis. The prognostic model was defined as follows: risk score = coefficient 1∗expression of paired lncRNA 1 + ⋯+coefficient n∗expression of paired lncRNA n. Risk score was transformed to *z*-score, and *z* − score = 0 was set as a cut-off to classify samples into high-risk and low-risk groups. Finally, receiver operating characteristic (ROC) curve in timeROC R package was used to analyze the effectiveness of the prognostic model.

## 3. Results

### 3.1. Identification of Two Molecular Subtypes Based on Immune-Related Paired lncRNAs

Immune-related lncRNAs were screened by the Pearson correlation analysis between expression of immune-related genes and lncRNAs. 42 immune-related lncRNAs and 332 immune-related genes were identified when correlation coefficient > 0.4 and FDR < 0.05. Then, 42 immune-related lncRNAs were loop-paired and 375-paired lncRNAs were generated. Using univariate Cox regression analysis in TARGET dataset, we obtained 26-paired lncRNAs correlated with osteosarcoma prognosis (*p* < 0.05). Based on the expression of 26-paired lncRNAs, consensus clustering was applied to cluster 84 osteosarcoma samples (Supplementary Table 1). The samples were neatly classified into two clusters when *k* = 2 (Figure 2(a)), with C1 group showing a more favorable overall survival than C2 group (*p* = 0.0013, Figure 2(b)). We observed higher T cell CD4 naive and plasma cell infiltration in the C2 subtype (Figure 2(c)).

### 3.2. Enrichment Analysis of KEGG Pathways and GO Function for DEGs of C1 and C2

As significantly differential prognosis was observed between C1 and C2, we examined the difference of expression feature between the two subtypes. 213 DEGs were screened between C1 and C2 when |FC| > 1.5 and *p* < 0.05. Specifically, 99 DEGs were downregulated and 114 DEGs were upregulated in C1 group. Enrichment analysis of KEGG pathways and GO function identified 240 terms of biological process, 15 terms of cellular component, 14 terms of molecular function, and 14 terms of functional pathways from the upregulated genes (*p* < 0.05). The top 10 terms of each column were visualized in Figure 3. Of the downregulated genes, 39 terms of biological process, 30 terms of cellular component, 5 terms of molecular function, and 2 KEGG pathways were annotated (*p* < 0.05, Figure 4). Terms of complement activation, inflammatory response, and immune response were greatly enriched in upregulated genes, suggesting an active immune response in C1 group (Figure 3(a)). Meanwhile, ECM-receptor interaction pathway potentially involved in cancer development was highly enriched in the downregulated genes that were highly expressed in C2 group (Figure 4(d)). These functional annotations validated the differential prognosis of two molecular subtypes.

### 3.3. The Difference of Tumor Microenvironment between the Two Molecular Subtypes

TME is consisted of various immune cells, tumor cells, stromal cells, cytokines, chemokines, and so on and can decide the progression of tumor cells. To understand the difference of TME between the two subtypes, ssGSEA was conducted to calculate the score of 22 immune cells of each sample, and we found an obviously higher enrichment of activated CD8 T cells, immature B cells, macrophages, myeloid derived suppressor cells (MDSCs), and regulator T cells in C1 group (Supplementary Figure S1A). In addition, we analyzed the expression of 13 immune metagenes identified by previous studies through ssGSEA [22, 29]. Each of the immune metagene contained a series genes related to immune response. The majority of metagenes were found to be highly expressed in C1 group, especially costimulation, cytolytic, immune score, and STAT1 (*p* < 0.05, Figure5(a)), which indicated higher immune response of C1 group. Similarly, ESTIMATE analysis also revealed higher immune score in C1 group (*p* = 0.033, Figure 5(b)). Furthermore, we included 47 immune checkpoints and compared their expression level between C1 and C2 groups. Only 7 immune checkpoints, including CD40, CD40LG, CD48, HAVCR2, LAG3, LAIR1, and TNFRSF4, presented significant difference between them (*p* < 0.05, Supplementary Figure S1B).

### 3.4. Sensitivity to Four Chemotherapeutic Drugs

We also assessed whether two molecular subtypes had different sensitivities to chemotherapeutic drugs. Four drugs of TAE684, BI-2536, A-443654, and GW843682X were used. The result exhibited that C2 group had lower estimated IC50 of four drugs than C1 group, indicating that C2 group was more sensitive to these drugs (*p* < 0.05, Figure 6). The finding suggested that patients with C2 subtype could benefit much from chemotherapy.

### 3.5. Construction of a 4-Paired lncRNA Prognostic Model

A sum of 84 osteosarcoma samples were divided into training cohort and test cohort with ratio 1 : 1 through random sampling. In the training cohort, 21-paired lncRNAs associated with prognosis were screened from 375-paired lncRNAs by univariate Cox regression analysis (*p* < 0.05). As a 21-paired lncRNA prognostic model was complex to apply in clinical practice, therefore, we performed LASSO and AIC to further simplify the model. LASSO regression analysis can reduce variables by introducing the lambda value. When lambda = 0.0506, the optimal model containing 8-paired lncRNAs was generated (Figure 7). Through utilizing stepAIC, a minimum number of variables can be obtained with considerable fitting degree. Finally, 4-paired lncRNAs were remained, and the prognostic model was defined as follows:

(1) $$\begin{array}{c} \text{Risk score}=-1.431*\left(\text{GOLGA}8\text{M vs}.\text{AJ}239318.1\right)-1.699*\left(\text{C}11\text{orf}44\text{ vs}.\text{C}1\text{orf}137\right)-1.593*\left(\text{FAM}215\text{A vs}.\text{C}1\text{orf}137\right)+1.755*\left(\text{SFTA}3\text{ vs}.\text{SPATA}8\right). \end{array}$$

Risk score was converted to *z*-score, and *z* − score = 0 was defined as a cut-off for classifying samples into high-risk (*z* − score > 0) and low-risk (*z* − score < 0) groups. In the training cohort, 22 samples were classified into high-risk group, and 20 samples were classified into low-risk group, with a distinct overall survival (*p* = 0.0017, Figure 8(a)). ROC analysis showed the effectiveness of the model in predicting 1-year, 3-year, and 5-year overall survival (Figure 8(b)). The robustness of the prognostic model was validated in the test cohort. Consistently, 42 samples were classified into high-risk and low-risk groups that were significantly with differential prognosis (*p* = 0.044, Supplementary Figure S2). Moreover, the tendency of survival status and expression of 4-paired lncRNAs changed consistently with the variation of risk score (Figure 9). The samples of dead status were more concentrated in the high-risk group. The expression level of FAM215A vs. C1orf137 and C11orf44 vs. C1orf137 paired lncRNAs were higher in the low-risk group.

In the relation of risk score to clinical features and molecular subtypes, we assessed their distribution in the high-risk and low-risk groups. The dead samples showed significant higher risk score than samples of alive status (Supplementary Figure S3A). The female and male samples had a similar distribution of risk score (Supplementary Figure S3B). Two molecular subtypes identified by the previous section displayed a significant difference in risk score (Supplementary Figure S3C). C2 subtype had higher risk score than C1 subtype, which was consistent with the poor survival of C2 subtype.

We systematically compared the relationship between the expression of GOLGA8M, AJ239318.1, C11orf44, C1orf137, FAM215A, SFTA3, and SPATA8 in paired lncRNAs and disease. We observed that GOLGA8M, C1orf137, and SFTA3 in these lncRNAs were significantly overexpressed in tumor samples (Supplementary Figure S4A). In addition, C11orf44 was significantly overexpressed in C1 subgroup, and C1orf137 was significantly overexpressed in C2 subgroup (Supplementary Figure S4B). Univariate and multivariate survival analyses showed that AJ239318.1 high expression was significantly correlated with poor prognosis (Supplementary Figure S4C-D). The scores of the 22 immune cells in each sample were calculated by CIBERSORT algorithm, and then, the correlation between the expression of these 7 lncRNAs and immune infiltration score was calculated by Pearson's method. It can be observed that T cell CD4 naïve, T cell CD4 memory resting, and T cell CD4 memory activated showed a significant positive correlation with C11orf44, C1orf137, FAM215A, and SFTA3 (Supplementary Figure S4E).

### 3.6. Identification and Functional Analysis of Genes Related to Four Prognostic Paired lncRNAs

To assess the possible function of these four-paired lncRNAs, Spearman's correlation analysis was performed to analyze the relation between lncRNAs and mRNAs. 661 genes were identified with a condition of correlation coefficient > 0.3 and *p* < 0.05. Then, we applied WebGestalt R package to annotate KEGG pathways and GO function significantly associated with 661 genes. The analysis showed 109 terms of biological process, 120 terms of cellular component, and 70 terms of molecular function (Figures 10(a)–10(c)). Calcium signaling pathway and cAMP signaling pathway involved in cancer development were annotated (Figure 10(d)).

## 4. Discussion

Previous studies have confirmed the essential role of lncRNAs in cancer cell proliferation, invasion, and metastasis. Aberrantly expressed lncRNAs secreted from cancer cells can help the cells escape from immune capture and create tumor-supportive immune microenvironment through the interactions with oncogenic pathways [18]. In osteosarcoma, low immune infiltration is shown in TME compared with other cancers, which may be the major reason leading to unsatisfactory results of immunotherapy [6–8]. The role of lncRNAs in shaping TME beneficial and facilitating tumor growth has not been completely understood. This study systematically examined and interpreted the close correlations among lncRNAs, TME, and prognosis, according to the transcriptional data of osteosarcoma samples and integrated bioinformatics analysis.

Compared with the absolute quantification based on gene expression profile, the relative ranking method has the advantages of independent standardization method and cross platform comparison. In this study, a new data matrix is established by using the relative rank of lncRNA. Using a paired lncRNA strategy and unsupervised consensus clustering, we identified two immune subtypes (C1 and C2) significantly associated with prognosis. Between the two subtypes, 213 differentially expressed immune-related genes contained 114 upregulated genes and 99 downregulated genes in C1. The functional analysis of these genes showed that the upregulated genes were enriched in the processes of immune response and inflammatory response and downregulated genes were enriched in ECM-receptor interaction pathway (Figures 3 and 4). Active immune response creates a condition for impeding the proliferation of cancer cells, which was consistent with the favorable prognosis of C1 subtype.

Extracellular matrix (ECM) can be deformed by proliferation of cancer cells and activation of fibroblasts in tumor, thereby resulting in vessel compression [30, 31]. Compressed vessels can hinder the transportation of immune cells to tumor site, hence promoting tumor growth and invasion [30]. ECM-receptor interaction pathway is more active in C2 subtype, which corresponds to its poorer overall survival. Studies have also demonstrated that ECM-related genes are upregulated in other cancer types such as prostate cancer and gastric cancer [32, 33]. In addition, ECM can interact with tumor-associated macrophages (TAMs) to regulate tumor angiogenesis and foster immunosuppressive microenvironment [34]. In an anti-VEGF therapy of colorectal cancer, ECM is remodeled and treatment efficacy is improved in mouse models [35]. Therefore, 26-paired lncRNAs significantly related to osteosarcoma prognosis may serve as key regulators for up- or downregulated expression of DEGs. ECM and ECM-receptor interaction pathway may be potential targets for cancer therapies of osteosarcoma.

In the relation between immune subtypes and TME, we observed higher immune infiltration in C1 subtype, which was majorly resulted from the higher enrichment of CD56 bright natural kill cells, immature B cells, macrophages, MDSCs, and regulatory T cells (Supplementary Figure S1). Analysis on immune-related genes also revealed a higher immune score in C1 subtype, especially metagenes of cytolytic activity (CYT) and STAT1 (Figure 5(a)). Perforin 1 (PRF1) and oxins granzyme A (GZMA) released by cytotoxic T cells and NK cells were used to calculate CYT score and reflect antitumor immunity in cancers [36]. High CYT score has been considered as a protective factor of the prognosis in many cancer types, such as hepatocellular carcinoma [37] and gastric cancer [38]. Moreover, the CYT score was positively associated with the expression of immune checkpoint molecules in prostate cancer [39] and colorectal cancer [40]. Higher expression of immune checkpoint molecules, particularly CD40, CD48, HAVCR2, LAG3, LGALS9, and TNFRSF4, was also found in C1 subtype (Supplementary Figure S1B), indicating that C1 could benefit much from immune checkpoint blockade. J. Zhang et al. found that anti-CD40 mAb treatment could enhance the efficacy of anti-PD-1 treatment through converting PD-1^hi^ T cells to PD-1^lo^ T cells [41]. It provides a possibility that these differentially expressed immune checkpoint molecules may be the therapeutic target for combined immunotherapies in osteosarcoma, especially C1 subtype.

Signal transducer and activator of transcription-1 (STAT1), which is regulated by lncRNA NEAT1, are involved in osteosarcoma metastasis [42]. The inhibition of STAT1 expression can activate EMT process of osteosarcoma sites [42]. In other cancer types, upregulated expression of STAT1 is also associated with favorable outcome [43, 44]. In our results, C1 subtype has a higher enrichment score of STAT1 and a better prognosis than C2 subtype, which was consistent with other studies. A number of lncRNAs such as PSMB8-AS1 [45], LINC01123 [46], and LINC00174 [47] interacting with STAT1 have been found to contribute tumor progression. The 26-paired lncRNAs identified in this study may also be involved in the interactions with STAT1 expression, which can serve as a basis to further examine STAT1 mechanism in cancer metastasis in the future study.

Two immune subtypes classified by different expression patterns of lncRNAs manifested differences in prognosis and TME and therefore further supported the critical role of lncRNAs in suppressing or promoting tumor growth and metastasis. Furthermore, the two subtypes provided a direction for developing new targeted immunotherapies and guiding the personalized application of four chemotherapeutic drugs.

Based on the 26-paired lncRNAs, we constructed a prognostic model with robust performance to predict prognosis of osteosarcoma patients. Patients were clearly stratified into high-risk and low-risk groups according to the expression of four-paired lncRNAs (GOLGA8M vs. AJ239318.1, C11orf44 vs. C1orf137, FAM215A vs. C1orf137, and SFTA3 vs. SPATA8). This 4-paired lncRNA signature enables a quick identification of patients with poor prognosis and promotes earlier treatment to avoid unfavorable outcomes. However, before the application of immune subtypes and prognostic signature, more clinical objects should be included to validate our results.

## 5. Conclusion

In conclusion, this study established an association among immune-related lncRNAs, TME, and osteosarcoma prognosis through identifying two immune subtypes and four-paired prognostic lncRNAs. We revealed that the ECM-receptor interaction pathway was a new therapeutic target for treating osteosarcoma patients. A possible relation was identified between CYT and immune checkpoints that could direct the personalized immunotherapy but requires further validation. The current findings showed the mechanism and role of lncRNAs in osteosarcoma progression such as the involvement of STAT1 interacting with lncRNAs. Importantly, the immune subtypes and 4-paired lncRNA signature could be useful tools in clinical practice.

## Figures and Tables

**Figure 1:** The workflow of constructing a prognostic model based on immune-related lncRNAs.

**Figure 2:** Consensus clustering for identifying two molecular subtypes. (a) Consensus matrix when cluster number *k* = 2. (b) The Kaplan-Meier survival curve of C1 and C2 subtypes. Log-rank test was performed. (c) Distribution difference of immune infiltrating cells in 22 of C1 and C2 subtypes.

**Figure 3:** Enrichment analysis of biological process (a), cellular component (b), molecular function (c), and KEGG pathways (d) in upregulated genes. The top 10 enriched terms were displayed. Vertical axis displays the annotated terms. Dot represents the counts of enriched genes in one term.

**Figure 4:** Enrichment analysis of biological process (a), cellular component (b), molecular function (c), and KEGG pathways (d) in downregulated genes. The top 10 enriched terms were displayed. Vertical axis displays the annotated terms. Dot represents the counts of enriched genes in one term.

**Figure 5:** The enrichment score of two molecular subtypes in 13 immune metagenes (a) and immune score (b). Student's *t* test was performed in 13 immune metagenes. The Kruskal-Wallis test was performed in immune score. ∗*p* < 0.05. ns: no significance.

**Figure 6:** The estimated IC50 of TAE684 (a), BI-2536 (b), A-443654 (c), and GW843682X (d) in C1 and C2 subtypes. The Wilcoxon test was performed.

**Figure 7:** LASSO Cox regression for 21-paired lncRNAs. (a) The track plot of 21-paired lncRNAs changing with the lambda value. Different colors of curves represent different paired lncRNAs. Red-dotted line represents the site of lambda = 0.0506. (b) The confidence interval of partial likelihood deviance changing with the lambda value. The orange dot represents the site of lambda = 0.0506.

**Figure 8:** The performance of 4-paired lncRNA prognostic model in the training cohort. (a) The Kaplan-Meier survival plot of high-risk and low-risk groups. Red curve represents high-risk group and dark blue represents low-risk group. Log-rank test was performed. (b) ROC curve of 1-year (red), 3-year (green), and 5-year (blue) overall survival.

**Figure 9:** The distribution of survival status and expression of four-paired lncRNAs corresponding with the risk score.

**Figure 10:** Enrichment analysis of biological process (a), cellular component (b), molecular function (c), and KEGG pathways (d) for 661 genes. The top 10 enriched terms were displayed. Vertical axis displays the annotated terms. Dot represents the counts of enriched genes in one term.

## Data Availability

The data used to support the findings of this study are included within the article.

## Supplementary Materials

Supplementary 1 Supplementary Figure S1: the enrichment score of 22 immune cells (A) and the log2 (gene expression+1) of 47 immune checkpoints (B) in two molecular subtypes.

Supplementary 2 Supplementary Figure S2: the performance of 4-paired lncRNA prognostic model in the test cohort. (A) The Kaplan-Meier survival plot of high-risk and low-risk groups. Red curve represents high-risk group and dark blue represents low-risk group. Log-rank test was performed. (B) ROC curve of 1-year (red), 3-year (green), and 5-year (blue) overall survival.

Supplementary 3 Supplementary Figure S3: the distribution of high-risk and low-risk samples in different survival status (A), genders (B), and molecular subtypes (C).

Supplementary 4 Supplementary Figure S4: the relationship between the expression of seven lncRNAs in paired lncRNAs and diseases. (A) The expression of seven lncRNAs was different between tumor and normal samples. (B) The expression differences of seven lncRNAs in C1 and C2 subtypes. (C) Univariate survival analysis showed the relationship between the expression of seven lncRNAs and prognosis. (D) Multivariate survival analysis showed the relationship between the expression of seven lncRNAs and prognosis. (E) Pearson correlation heatmap between the expression of 7 lncRNAs and 22 immune cell infiltration scores.

Supplementary 5 Supplementary Table 1: molecular subtype information of each sample.
